The article "Determination of Genetic and Epigenetic Modifications-Related Prognostic Biomarkers of Breast Cancer: Genome High-Throughput Data Analysis" was published in 2021. Journal: J Oncol.

# Determination of Genetic and Epigenetic Modifications-Related Prognostic Biomarkers of Breast Cancer: Genome High-Throughput Data Analysis

**DOI:** 10.1155/2021/2143362

**Published:** 2021-09-13

**Authors:** Chundi Gao, Huayao Li, Cun Liu, Jibiao Wu, Chao Zhou, Lijuan Liu, Jing Zhuang, Changgang Sun

**Affiliations:** ^1^College of First Clinical Medicine, Shandong University of Traditional Chinese Medicine, Jinan, Shandong 250014, China; ^2^College of Basic Medical, Shandong University of Traditional Chinese Medicine, Jinan, Shandong 250014, China; ^3^Department of Oncology, Weifang Traditional Chinese Hospital, Weifang, Shandong 261041, China; ^4^Qingdao Academy of Chinese Medical Sciences, Shandong University of Traditional Chinese Medicine, Qingdao, China

## Abstract

The high heterogeneity of breast cancer (BRCA) makes it more challenging to interpret the genetic variation mechanisms involved in BRCA pathogenesis and prognosis. Areas with high DNA methylation (such as CpG islands) were accompanied by copy number variation (CNV), and these genomic variations affected the level of DNA methylation. In this study, we characterized intertumor heterogeneity and analyzed the effects of CNV on DNA methylation and gene expression. In addition, we performed a Genetic Set Enrichment Analysis (GSEA) to identify key pathways for changes between patients with low and high expression of genes. Our analysis found two key genes, namely, HPDL and SOX17. The protein expressed by HPDL is 4-hydroxyphenylpyruvate dioxygenase-like protein, which has dioxygenase activity. SOX17 is a transcription factor that can inhibit Wnt signaling, promote the degradation of activated CTNNB1, and participate in cell proliferation. Our analysis found that the CNV of HPDL and SOX17 is not only related to the patient's prognosis, but also related to gene methylation and expression levels affecting the patient's survival time. Among them, the high-methylation, low-expression HPDL and SOX17 showed poor prognosis. And the addition of two copies of SOX17 is associated with a lower survival rate, while a decrease in the copy number of HPDL also suggests a poor prognosis. This study provided an effective bioinformatics basis for further exploration of molecular mechanisms related to BRCA and assessment of patient prognosis, but the development of biomarkers for diagnosis and treatment still requires further clinical data validation.

## 1. Introduction 

In the postgenomic era, rapidly evolving high-throughput sequencing technologies have enabled the acquisition of vast amounts of multiomics data more efficiently [1]. The variation of expression of some genes causes the genetic regulation trajectory inside the cell to deviate, which alters the gene expression programming inside the cell. Therefore, most disease-causing genomic variants are likely to play a role by altering gene regulation, such as transcription factor binding and DNA methylation, rather than directly affecting protein function [2, 3]. The high heterogeneity of breast cancer (BRCA) makes it more challenging to interpret the genetic variation mechanisms involved in BRCA pathogenesis and prognosis [4].

In human cancer, genomic instability leads to extensive cell copy number variation (CNV) [5]. Genome-wide association studies (GWASs) have been conducted for common malignancies and have identified more than 450 genetic variants associated with increased disease risk [6]. In BRCA, CNV is associated with about 40% of gene expression, which can participate in the occurrence and development of BRCA and affect the prognosis of patients [7]. It has been found that changes in CNV such as BRCA1, BLM, and OR4C11 will increase the incidence of BRCA. BRCA1, BLM, and OR4C11 are all related to cell proliferation. BRCA1 is a transcriptional activator that can regulate the cell cycle; BLM is involved in DNA replication and repair, and OR4C11 can regulate cell signal transduction [8], while changes in CNV such as MYC and JAK2 play a role in acquired chemotherapy resistance to triple-negative BRCA [9]. In addition, the higher intratumoral heterogeneity of EGFR/CEP7 and CCND1/CEP11 CNV could predict metastasis and was significantly correlated with metastasis-free survival in triple negative BRCA patients [10].

Disorders in the epigenetic state are closely related to human diseases, particularly cancer. DNA methylation is a well-characterized epigenetic modification that is closely related to many cellular processes. In the current study, DNA methylation and its sites associated with tumor recurrence and overall survival (OS) of BRCA and its subtypes have been identified based on methods employed for genome-wide DNA methylation analysis [11–13]. The methylation of oncogenes, ESR1 and ERBB2, and tumor suppressor genes, FBLN2, CEBPA, and FAT4, contribute to the early diagnosis of BRCA [14]. And the methylation of HER2, Ki67, and GSTP1 are associated with BRCA TNM staging and tumor size and can be combined for early diagnosis and prognosis [15].

CNV represents a major source of genomic variation and is an important genetic factor leading to various cancers. DNA methylation, a major means of epigenetic modification, is considered an inhibitory epigenetic marker. Several studies have found that areas with high DNA methylation (such as CpG islands) are accompanied by copy number variation, and these genomic variations affect the level of DNA methylation [16]. For example, in lung adenocarcinoma, DNA methylation heterogeneity demonstrates branch clonal evolution of lung adenocarcinoma regions driven by genomic instability and subclone copy number variation [17]. Here, we investigated the association between genomic variation (such as CNV) in regulatory regions of BRCA and corresponding changes in DNA methylation. In addition, we performed a Genetic Set Enrichment Analysis (GSEA) to identify key pathways for changes between patients with low and high expression of genes. Thus, an in-depth study of the genome pathogenesis of BRCA was conducted to identify prognostic biomarkers and their clinical efficiency.

## 2. Materials and Methods

### 2.1. Data Processing and Analysis

The BRCA-related methylation, CNV, gene expression, and clinical data were downloaded from The Cancer Genome Atlas (TCGA) GDC (https://gdc.cancer.gov/). The chi-square test and Limma and edgeR software packages were used to collate and analyze the downloaded data and screened according to *P* and logFC values. To obtain differences in CNV, abnormally methylated and dysregulated genes between BRCA tissue samples and normal tissue samples were analyzed. The data from the TCGA database is public. Therefore, no approval from the local ethics committee was required.

### 2.2. Multilayer Correlation Analysis Predicts the Pattern of Gene CNV in BRCA

DNA methylation has been shown to regulate gene expression in a variety of ways, such as changing chromosome structure, DNA stability, etc. In addition, CNV is widely distributed in the human genome and has important biological implications. To further explore the link between CNV and methylation on gene expression, the possible patterns of CNV in BRCA need to be elucidated. This study focuses on the analysis of correlation between abnormal methylation and gene expression, CNV and aberrant methylation, and CNV and gene expression. Screening was done by the Pearson correlation coefficient and *P* value. Key genes with simultaneous methylation abnormalities, CNV, and abnormal expression were obtained, and further prognostic analysis was performed on these genes.

### 2.3. Mapping of Kaplan–Meier Survival Curve of Genes and Screening of Prognostic Key Genes

In order to further identify key genes related to the prognosis of BRCA patients from the genes obtained above, survival analysis was performed on the relevant data based on the survival software package, and survival curves were plotted to show the effect of abnormal methylation and methylation combined with abnormal gene expression on patient survival. In addition, in order to further explore the methylation sites of prognostic aberrant methylation genes, the factors affecting the prognosis of patients and gene expression are mapped to specific methylation sites.

### 2.4. The Impact of CNV of Key Genes on Patient Prognosis

Through data analysis, it was found that the abnormal methylation of key genes is closely related to the prognosis of BRCA patients, while the key genes harbored methylation abnormalities, CNV, and abnormal expression, and there was a significant correlation between them. The effect of mutations on the prognosis of patients can be seen by studying CNV and survival time of BRCA patients, further indicating the biological significance of gene CNV in the progression of BRCA. In addition, we performed GSEA analysis between high-expression and low-expression groups of key genes to determine key pathways that are altered in patients with abnormal gene expression [18].

## 3. Results

### 3.1. Data Processing and Analysis

In this study, BRCA-related methylation data downloaded from the TCGA database included 883 samples, comprising 96 normal tissue samples and 787 BRCA tissue samples. The difference analysis results obtained a total of 122 protein-coding genes with *P* < 0.05 and |logFC| > 1 as the cutoff condition (Figure 1(a)). The CNV data included 2201 samples, 1103 normal tissue samples, and 1098 BRCA tissue samples. A total of 19178 genes with CNV were found based on the chi-square test results (*P* < 0.05) (Supplementary Material 1). The difference analysis of gene expression data between 112 normal tissue samples and 1096 cancer tissue samples showed that 2138 dysregulated genes, including 1375 upregulated genes and 763 down regulated genes (Figure 1(b)), were obtained with *P* < 0.01 and |logFC| > 2 as the cutoff condition.

### 3.2. Multilayer Correlation Analysis to Screen Key Genes

In order to reduce the number of calculations of correlation analysis between the two, we performed correlation analysis on the condition of genes with abnormal methylation. First, we found that 105 of the 122 genes with aberrant methylation exhibited simultaneous expression disorders. Combining methylation and expression-related samples (857 in total) for correlation analysis showed that the aberrant methylation of 25 genes was closely related to the expression with the Pearson correlation coefficient Cor  > 0.4 as the screening criterion (Table 1). Interestingly, these 25 genes harbored CNV simultaneously (Figure 1(c)). To explore the pattern of effects of CNV in disease progression, we performed a correlation analysis of CNV with methylation and abnormal gene expression for 25 genes. Among them, CNV and methylation-related samples were combined with a total of 855, and CNV and expression-related samples were combined with a total of 1172. Screening with *P* < 0.01 as the cut-off criterion, the CNV of 12 genes was associated with the level of methylation, and the CNV of 16 genes was related to the abnormal expression level. Among them, there are 6 common genes (Figure 2). We used these six genes as key genes for prognostic survival analysis.

### 3.3. Joint Survival Analysis and Site-Related Prognostic Assessment to Identify Biomarkers

Through joint survival analysis, it was found that the combination of methylation and abnormal expression of HPDL and SOX17 was significantly associated with the prognosis of BRCA patients. Furthermore, the results showed that high-methylation low-expression of HPDL and SOX17 showed poor prognosis (Figure 3(a)). In addition, based on the survival of the R package, we analyzed the effects of the relevant methylation sites of these two genes on patient survival. *P* < 0.05 was used as a screening criterion for predicting prognosis, and specific methylation sites associated with the prognosis of these genes were found. Among them, the two methylation sites of HPDL and the eight methylation sites of SOX17 can affect the survival time of patients (Figure 3(b)).

### 3.4. Kaplan–Meier Survival Curve Analysis of the Effect of Gene CNV on Patient Prognosis

The genes HPDL and SOX17 showed not only methylation abnormalities and abnormal expression, but also CNV. Further analysis showed that CNV in HPDL and SOX17 were associated with overall patient survival, in which the addition of two copies of SOX17 is associated with a lower survival rate, while a decrease in the copy number of HPDL also suggests a poor prognosis (Figure 3(c)). In addition, as the CNV of HPDL and SOX17 are related to methylation and abnormal expression levels, our research indicated that the CNV of HPDL and SOX17 can directly affect the prognosis of patients and can also indirectly affect the survival time of patients by affecting the methylation and expression levels of the corresponding genes.

### 3.5. GSEA Analysis of Patients with Low and High Expression of HPDL and SOX17

To identify the molecular pathways of the biological functions and effects of HPDL and SOX17 in BRCA progression, we used GSEA to identify key pathways involved in the changes between patients with low and high expression of genes. With *P* value < 0.05 as the screening standard, the results indicated that the pathways that HPDL can affect mainly, including MAPK signaling pathway and p53 signaling pathway. In addition, SOX17 mainly affects JAK-STAT signaling pathway, WNT signaling pathway, and so on (Table 2, Figure 4).

## 4. Discussion

Heterogeneity is an important predictor of tumor treatment failure and drug resistance, and genomic mutations (such as copy number variation) are important causal factors of heterogeneity among tumors. Previous studies have shown that CNV can affect the expression level of proteins through epigenetic regulation, and the key mechanism is to affect epigenetic modifications (such as DNA methylation). The overall hypomethylation of oncogenes and hypermethylation of tumor suppressor genes are characteristic of most cancer types. Molecular understanding of BRCA heterogeneity is the key to effective treatment and personalized medicine. In this study, we used TCGA high-throughput molecular profiling data to characterize intertumor heterogeneity and analyzed the effects of CNV on DNA methylation and gene expression.

In our analysis, CNV of HPDL and SOX17 affected methylation and gene expression levels in BRCA, and CNV and methylation of HPDL and SOX17 can lead to poor prognosis in patients with BRCA. In this study, it was found that the CNV of SOX17 showed copy number amplification on chromosome 8, while the CNV of HPDL showed a decrease in copy number on chromosome 1. Further analysis showed that when the copy number of SOX17 increased or the copy number of HPDL decreased, the prognosis of BRCA patients was poor. The CNV of SOX17 and HPDL can affect the expression of genes through epigenetic modification, and DNA methylation is an important pathway for epigenetic modification. The methylation sites of SOX17 that we characterized with BRCA OS included cg00123055, cg02222728, cg03329976, cg08044907, cg15377283, cg24150172, cg24891539, and cg24928317. The methylation sites of HPDL included cg12178578 and cg15071854. Survival analysis showed that the OS of BRCA patients hypermethylated in SOX17 and HPDL was poorer. Therefore, CNV and methylation of SOX17 and HPDL could predict recurrence, metastasis, and prognosis of BRCA patients.

SOX17, a transcriptional regulator, binds to target promoter DNA and inhibits Wnt signaling. SOX17 gene promoter methylation can be used as a tumor suppressor and dysregulated oncogene in many tumors [19–21]. In BRCA, Fu et al. used methylation-specific polymerase chain reaction to assess the relationship between the methylation of the SOX17 gene promoter and the onset and prognosis of BRCA. Abnormal SOX17 methylation in cancer tissues and plasma DNA was found to be significantly associated with tumor lymph node metastasis and lymph node metastasis, associated with poor disease-free survival (*P* < 0.005) and overall survival (*P* < 0.005). In addition, SOX17 methylation in plasma DNA is an independent prognostic factor for DFS in BRCA [22]. Chimonidou et al. found that the SOX17 promoter is highly methylated in primary breast tumors, in CTCs isolated from patients with BRCA, and in corresponding cfDNA samples, which provides new predictive ideas for recurrence and prognosis in patients with operable BRCA and metastatic patients [23, 24]. HPDL may have dioxygenase activity. Previous studies have found that HPDL exhibits differential expression in CNS lymphoma compared with nonprimary central nervous system (CNS) lymphoma [25]. However, understanding the role of HPDL in BRCA needs further research and interpretation, which provides an idea for the in-depth study of the molecular mechanism of BRCA.

Intracellular signaling pathways regulate various cellular activities. We performed GSEA identification on SOX17 and HPDL to further explore the small-molecule regulation mechanism of BRCA and found that signaling pathways with significant changes in enrichment exist between patients with low expression and high expression. When SOX17 is downregulated, the enriched pathways mainly included JAK-STAT signaling pathway and Wnt signaling pathway. It is well known that the JAK-STAT signaling pathway, a signal transduction pathway stimulated by cytokines, is involved in biological processes, such as cell proliferation, differentiation, apoptosis, and immune regulation, and is associated with pathogenesis of many tumors, such as liver cancer, ovarian cancer, and BRCA [26–28]. The major cellular processes during BRCA development rely on JAK/STAT signaling to coordinate growth factor function. Previous studies have found that activation of the JAK/STAT pathway is common in triple-negative BRCA, which can affect the expression of genes controlling immune signals. Dysregulated JAK/STAT signaling has been implicated in BRCA metastasis, associated with high risk of recurrence [29–31]. The Wnt signaling pathway plays a crucial role in early embryonic development, organ formation, tissue regeneration, and other physiological processes, often involving stem cell control, which may induce cancer if a key protein is mutated [32]. Wnt signaling pathway involves the onset and treatment of colorectal cancer, pancreatic cancer, gastric cancer, and other tumors [33–35]. Yang et al. confirmed that SOX17 is a target gene of miR-194-5p. In mouse studies, knockdown of miR-194-5p in BRCA cells may increase SOX17 expression and regulate the signaling pathway of Wnt/*β*-catenin [36]. Therefore, increased expression of SOX17 can activate the Wnt signaling pathway and, thus, participate in the pathogenesis of BRCA. In addition, the enrichment results of SOX17 include pathways related to cell growth, division, and proliferation of oocyte meiosis, ABC transporters, and neuroactive ligand-receptor interaction.

The enrichment pathways of HPDL upregulation mainly include cell cycle and P53 signaling pathway. And the HPDL downregulation is mainly enriched in MAPK signaling pathway and TGF-*β* signaling pathway. Both cell cycle and p53 signaling pathways are involved in cell division and proliferation. The p53 gene is called the “guardian of the genome,” but when p53 is deregulated, it participates in the development and proliferation of various tumor cells [37]. Both MAPK and TGF-*β* signaling pathway are involved in cell growth, differentiation, and apoptosis. In recent studies, abnormal activation of the MAPK signaling pathway signal has been found to favor the abnormal proliferation of malignant cells [38]. TGF-*β* signaling acts as suppressor and inducer of tumor progression during the early and late stages of cancer and can trigger a cascade of reactions that mobilize cancer cells [39, 40].

Recent studies have demonstrated the consequences of genetic variation in regulating overall risk associated with BRCA patients. In the study so far, we explored the effects of CNV and DNA methylation on gene expression levels and OS of BRCA patients and found that CNV can affect DNA methylation levels. CNV and methylation of SOX17 and HPDL are related to expression and regulation. In addition, the CNV of SOX17 and HPDL were also correlated with methylation levels. In addition, we found methylation sites for SOX17 and HPDL associated with BRCA prognosis. DNA methylation is an effective regulator of gene expression. If the CpG island is located in the promoter region of a gene, the methylation of the CpG island will significantly reduce or even completely silence the transcription of the gene and then affect the protein expression. In this study, due to data and conditional restrictions, we did not distinguish whether it was on the promoter or DNA when screening prognostic related methylation sites, which is what we will explore in the next study. Finally, by enriching the low and high expression pathways of SOX17 and HPDL, pathways related to BRCA progression have been discovered, including the JAK-STAT/Wnt/P53/MAPK signaling pathway.

However, this research also has certain limitations. For example, the quality of the samples in the TCGA database is very high, but the number of samples is very large. Therefore, the development of biomarkers for diagnosis and treatment still needs further clinical data verification. In future work, we will further increase the in-depth research and verification of our research results.

## 5. Conclusion

In summary, by comprehensively assessing the effects of CNV and DNA methylation on gene expression and patient OS, the CNV and DNA methylation associated with the risk of BRCA recurrence and prognosis were identified. These new discoveries are very promising. Prognostic assessment at the genome level may not only be useful for identifying new prognostic biomarkers, but would also open up new horizons for novel pathways involved in BRCA progression, serving the potential goal of developing more effective therapeutic strategies.

## Figures and Tables

**Figure 1:** (a) The heat map of BRCA-related aberrant methylated genes. The color from green to red shows a trend from low expression to high expression. (b) The volcano diagram of BRCA-related differentially expressed genes. The red dot represents upregulated genes, and green dot represents downregulated genes. (c) The CNV circle map of BRCA-related genes on chromosome. The points at the periphery indicate copy number amplification, and the points at the inner circumference indicate a decrease in copy number.

**Figure 2:** Six genes with CNV mutations that are related to both methylation and gene expression levels. (a–f) CNV and methylation. (g–l) CNV and expression.

**Figure 3:** (a) Kaplan–Meier survival curves for the joint survival analysis. (A) The combination of gene HPDL methylation and expression; (B) the combination of gene SOX17 methylation and expression. (b) Kaplan–Meier survival curves of the related methylated sites. (A, B) Methylated sites of the gene HPDL; (C–J) methylated sites of the gene SOX17. (c) Kaplan–Meier survival curves for the copy number variation.

**Figure 4:** Related pathways for abnormal expression of key genes in patients.

**Table 1:** 25 genes with significant correlation between methylation level and expression.

Gene	Cor	*P* value
HOXB13	0.455	5.47*E *− 45
SCGB3A1	−0.404	5.75*E *− 35
POU4F1	−0.411	2.76*E *− 36
SOX17	−0.412	2.06*E *− 36
SLC35G2	−0.417	2.56*E *− 37
RASSF10	−0.421	4.45*E *− 38
AADAT	−0.422	2.84*E *− 38
HFM1	−0.424	1.23*E *− 38
HPDL	−0.426	3.82*E *− 39
SNCA	−0.427	2.85*E *− 39
TBX18	−0.429	1.18*E *− 39
VIM	−0.475	1.99*E *− 49
DSC3	−0.503	4.94*E *− 56
LRRC34	−0.505	1.23*E *− 56
ZSCAN23	−0.53	2.24*E *− 63
ZNF454	−0.538	2.08*E *− 65
ZNF728	−0.545	1.39*E *− 67
MT1E	−0.566	9.90*E *− 74
IRX1	−0.567	4.62*E *− 74
ZNF492	−0.584	1.55*E *− 79
PSAT1	−0.587	1.64*E *− 80
EID3	−0.599	1.23*E *− 84
ID4	−0.605	1.26*E *− 86
HIST3H2A	−0.658	2.66*E *− 107
ZNF471	−0.662	3.79*E *− 109

**Table 2:** The key pathways for the differential between low and high expression of patients based on GSEA analysis.

Gene	Name	NES	*P* value
HPDL	KEGG_FOCAL_ADHESION	−1.91198	*P* < 0.001
	KEGG_DILATED_CARDIOMYOPATHY	−1.61559	0.002
	KEGG_HYPERTROPHIC_CARDIOMYOPATHY_HCM	−1.64029	0.002075
	KEGG_ADHERENS_JUNCTION	−1.74735	0.002283
	KEGG_ALDOSTERONE_REGULATED_SODIUM_REABSORPTION	−1.70915	0.002387
	KEGG_ARRHYTHMOGENIC_RIGHT_VENTRICULAR_CARDIOMYOPATHY_ARVC	−1.75006	0.006993
	KEGG_ABC_TRANSPORTERS	−1.5166	0.014141
	KEGG_MAPK_SIGNALING_PATHWAY	−1.66251	0.016713
	KEGG_TGF_BETA_SIGNALING_PATHWAY	−1.52333	0.04008
	KEGG_OOCYTE_MEIOSIS	1.754743	*P* < 0.001
	KEGG_PROGESTERONE_MEDIATED_OOCYTE_MATURATION	1.685132	*P* < 0.001
	KEGG_CELL_CYCLE	1.639552	*P* < 0.001
	KEGG_P53_SIGNALING_PATHWAY	1.51856	0.035503
	KEGG_OLFACTORY_TRANSDUCTION	1.609742	0.046472

SOX17	KEGG_OOCYTE_MEIOSIS	−1.58789	0.04814
	KEGG_JAK_STAT_SIGNALING_PATHWAY	1.797007	*P* < 0.001
	KEGG_NEUROACTIVE_LIGAND_RECEPTOR_INTERACTION	1.865758	0.001481
	KEGG_ABC_TRANSPORTERS	1.455277	0.014463
	KEGG_RETINOL_METABOLISM	1.741166	0.017483
	KEGG_HEMATOPOIETIC_CELL_LINEAGE	1.564893	0.021195
	KEGG_VASCULAR_SMOOTH_MUSCLE_CONTRACTION	1.562236	0.023636
	KEGG_ADIPOCYTOKINE_SIGNALING_PATHWAY	1.588887	0.029297
	KEGG_INSULIN_SIGNALING_PATHWAY	1.672106	0.038113
	KEGG_METABOLISM_OF_XENOBIOTICS_BY_CYTOCHROME_P450	1.663495	0.039587
	KEGG_WNT_SIGNALING_PATHWAY	1.528532	0.04
	KEGG_DRUG_METABOLISM_CYTOCHROME_P450	1.675274	0.043328
	KEGG_AXON_GUIDANCE	1.497392	0.047445

## Data Availability

The datasets generated and/or analyzed during the current study are available in the TCGA (https://cancergenome.nih.gov/).

## Abbreviations

BRCA: Breast cancer
CNV: Copy number variation
TCGA: The Cancer Genome Atlas
GSEA: Genetic Set Enrichment Analysis
OS: Overall survival.

## Supplementary Materials

Supplementary Materials Supplementary Material 1: genes with abnormal CNV mutations between breast cancer and normal tissues.
